# A New Variable-Censoring Control Chart Using Lifetime Performance Index under Exponential and Weibull Distributions

**DOI:** 10.1155/2021/1350169

**Published:** 2021-12-27

**Authors:** Muhammad Aslam, P. Jeyadurga, S. Balamurali, Rehan Ahmad Khan Sherwani, Mohammed Albassam, Chi-Hyuck Jun

**Affiliations:** ^1^Department of Statistics, Faculty of Science, King Abdulaziz University, Jeddah, Saudi Arabia; ^2^Department of Mathematics, Kalasalingam University, Krishnankoil 626126, Tamilnadu, India; ^3^College of Statistical and Actuarial Sciences, University of the Punjab, Lahore, Pakistan; ^4^Department of Industrial and Management Engineering, POSTECH, Pohang 37673, Republic of Korea

## Abstract

In reliability theory or life testing, exponential distribution and Weibull distribution are frequently considered to model the lifetime of the components or systems. In this paper, we design a control chart based on the lifetime performance index using Type II censoring for exponential and Weibull distributions. Average run length helps to measure the performance of the proposed control chart. The optimal values of the number of failure items and decision criteria used to decide whether the process is in-control or out-of-control based on the sample results are determined such that the in-control average run length is as close as to the specified average run length values. We simulate the data to illustrate the performance of the proposed control chart.

## 1. Introduction

In all production processes, the most important task for each manufacturer is to maintain the process stability because products with uniform quality can be achieved only when the process is stable. Process stability is defined as a state in which a process has shown a certain degree of consistency in history and is expected to continue the same state in the future. To maintain process stability, the cause of process variation should be detected and controlled because the process may be affected by either common causes or by assignable causes. Under this situation, the most important tool of statistical process control, namely, the control chart, helps the manufacturer. Specifically, a control chart is a graphical representation that shows the process variation over a period of time. Control charts can be used to achieve and maintain process stability via monitoring, analyzing, and understanding the process variations. There are two types of control charts available such as attribute control chart and variable control chart. The former is applicable where the quality characteristic of the sample is nonmeasurable, and the latter is used to monitor the measurable quality characteristic. One can find more applications of control charts in the production field (see, for example, Bersimis et al. [1]; Zhu et al. [2]; Chong et al. [3]; Jeyadurga et al. [4]; Ali et al. [5]). It is to be mentioned that statistical distributions play an important role in designing control charts. In particular, normal distribution was frequently used when designing variable control charts in earlier years. But, in recent years, numerous distributions such as exponential, Weibull, gamma, etc. are involved in designing control charts (see, for example, Aslam et al. [6, 7]; Ali and Pievatolo [8]; Ali et al. [5, 9]). In this study, we consider the designing of the control chart under exponential and Weibull distributions.

The lifetime is considered as the most essential characteristic of a product among other quality characteristics. For this reason, the producers concentrate on the lifetime of the products during the manufacturing process and a life test is conducted to determine the reliability of the products. However, the testing on the entire product is not possible due to time and cost constraints, whereas the test must be conducted to inspect the reliability. Under this situation, a time-censored life test (Type I) or failure-censored life test (Type II) is performed. In Type I censoring, the test termination time is prescribed in advance and it is observed that how many sample items failed until the time is attained. But, in Type II censoring, the number of failures is specified rather than the time. That is, the life test is terminated immediately if the specified number of failed items is attained. In this work, we consider Type II censoring in which a random sample of *n* items is placed in the life test and the test is terminated at the failure of the *s*^th^ sample item.

Process capability indices measure the ability of an in-control process to produce the products within the specification limits. One can obtain the relationship between the actual performance of the process and the specification limit by such measure. These indices are considered process improvement techniques. Similarly, Montgomery [10] introduced the lifetime performance index *C*_*L*_, which is utilized to evaluate the lifetime performance of a process with respect to a lower specification limit *L*. Some authors investigated the uniformly minimum variance unbiased estimator and hypothesis testing procedure of *C*_*L*_ under various distributions (see, for example, Tong et al. [11]; Wu et al. [12]; Lee et al. [13]; Lee et al. [14]; Lee et al. [15]; Lee [16]; Ahmadi et al. [17], Jafari and Bafekri [18]). In general, a normal distribution is considered as suitable to model the measurable quality characteristic of the products. But, the normal distribution is not appropriate to model the random variable that represents the time-to-failure (i.e., lifetime *T*) of electronic components since such random variable takes only positive values. In this circumstance, exponential or Weibull distribution is preferred as a suitable lifetime model rather than the normal distribution. Therefore, in this study, we consider exponential and Weibull distributions to evaluate the lifetime performance of a process. Numerous authors designed acceptance sampling plans using the lifetime performance index under exponential, gamma, and Weibull distributions (see, for example, Aslam et al. [19]; Wu et al. [20]; Lee et al. [21]). But, the study on designing control charts for exponential and Weibull distributions based on *C*_L_ under Type II censoring is not available in the literature. Therefore, we attempt to design such a control chart to monitor the lifetime performance of a process. The performance of the proposed control chart is measured by average run length (ARL) and is defined as the number of plotted points in the control chart before the out-of-control indication. In this work, the simultaneous minimization of out-of-control ARL and the number of failures to be observed under inspection are considered. The performance of the proposed control chart is explained by using simulated data.

## 2. Designing of the Control Chart under Lifetime Distributions

In this section, we discuss the designing of the control charts under exponential and Weibull distributions based on the lifetime performance index.

### 2.1. Designing of the Proposed Chart under Exponential Distribution

Suppose that the lifetime of the products is defined by the random variable *T* and *μ*_*T*_ and *σ*_*T*_ are the mean and standard deviation of lifetimes, respectively. The index *C*_*L*_ measures the performance of the process and is defined by (see Tong et al. [11])

(1) $$\begin{array}{c} C_{L}=\frac{\mu_{T}-L}{\sigma_{T}}, \end{array}$$

where *L* is a lower lifetime limit. Suppose that the random variable *T* follows an exponential distribution with parameter *λ* > 0 and have the probability density function (pdf) as follows:

(2) $$\begin{array}{c} f\left(t;\lambda \right)=\lambda e^{-\lambda t},\;t\geq 0. \end{array}$$

For exponential distribution, the mean and standard deviation are same. The exponential distribution with pdf given in equation (2) has mean 1/*λ* (i.e., *μ*_*T*_=1/*λ*) and standard deviation 1/*λ* (i.e., *σ*_*T*_=1/*λ*). Hence, by the substitution of *µ*_*T*_ and *σ*_*T*_ in equation (1), *C*_*L*_ can be simplified and rewritten as follows:

(3) $$\begin{array}{c} C_{L}=\frac{1/\lambda -L}{1/\lambda }=\frac{1/\lambda }{1/\lambda }-\frac{L}{1/\lambda }=1-\lambda L,\;-\infty <C_{L}<1. \end{array}$$

The lifetime-nonconforming rate is defined by

(4) $$\begin{array}{c} p=P\left(T\leq L\right)=1-e^{-\lambda L}=1-e^{C_{L}-1}. \end{array}$$

In practice, *λ* is usually unknown. In Type II censoring, *s* failures *t*_(1)_, *t*_(2)_,…, *t*_(*s*)_ are noted from *t*_(1)_, *t*_(2)_,…, *t*_(*n*)_. Wu et al. [20] provided the estimator of *λ* under Type II right censoring which is given by

(5) $$\begin{array}{c} {\hat{C}}_{L}=1-\hat{\lambda }L=1-\frac{\left(s-1\right)L}{\sum_{i=1}^{s}t_{\left(i\right)}+\left(n-s\right)t_{\left(s\right)}}. \end{array}$$

Suppose that *W*=∑_*i*=1_^*s*^*t*_(*i*)_+(*n* − *s*)*t*_(*s*)_. For this case, *s* is predefined so the statistic *W* is sufficient for *λ* which leads that 2*λW* follows a chi-squared distribution with 2*s* degrees of freedom (i.e., 2*λW* ~ *χ*_2*s*_^2^).

When designing a control chart under exponential and Weibull distributions, we need two parameters such as *H*_1_ and *H*_2_ instead of control limits used in traditional control charts. That is, instead of finding control limit coefficients in the traditional designing procedure, the optimal values of *H*_1_ and *H*_2_ are found so that the in-control ARL is as close as to the specified ARL and the statistic obtained from the process is compared with these optimal values of such parameters. Then, the process is said to be in-control if the statistic lies between *H*_1_ and *H*_2_; otherwise, the process is declared as out-of-control. The construction of the proposed control chart is as follows.

**Step 1 .**

Select a random sample of size *n* from the production process for the life test. Record first *s*(*n* ≥ *s*) failure times *t*_(1)_, *t*_(2)_,…, *t*_(*s*)_.

**Step 2 .**

Calculate ${\hat{C}}_{L}=1-\left(\left(s-1\right)L/\sum_{i=1}^{s}t_{\left(i\right)}+\left(n-s\right)t_{\left(s\right)}\right)$ (see Wu et al. [20]). Declare the process is out-of-control if either ${\hat{C}}_{L}\geq H_{2}$ or ${\hat{C}}_{L}\leq H_{1}$. Declare the process is in-control state if $H_{1}\leq {\hat{C}}_{L}\leq H_{2}$.

The probability that the process is to be declared as out-of-control is given by

(6) $$\begin{array}{c} P_{\text{out}}=P\left({\hat{C}}_{L}\geq H_{2}\right)+P\left({\hat{C}}_{L}\leq H_{1}\right)=1-P\left({\hat{C}}_{L}\geq H_{1}\right)+P\left({\hat{C}}_{L}\geq H_{2}\right),\\ P_{\text{out}}=1-P\left(1-\frac{\left(s-1\right)L}{\sum_{i=1}^{s}t_{\left(i\right)}+\left(n-s\right)t_{\left(s\right)}}\geq H_{1}\right)+P\left(1-\frac{\left(s-1\right)L}{\sum_{i=1}^{s}t_{\left(i\right)}+\left(n-s\right)t_{\left(s\right)}}\geq H_{2}\right). \end{array}$$

By following Wu et al. [20], *P*_out_ can be written as

(7) $$\begin{array}{c} P_{\text{out}}=1-P\left(\chi_{2s}^{2}\geq \frac{2\left(s-1\right)\left(1-C_{L}\right)}{\left(1-H_{1}\right)}\right)+P\left(\chi_{2s}^{2}\geq \frac{2\left(s-1\right)\left(1-C_{L}\right)}{\left(1-H_{2}\right)}\right). \end{array}$$

The probability that the process is declared to be out-of-control, when the process is at *C*_*L*_=*C*_*L*_^0^=1 − *λ*_0_*L*, is given by

(8) $$\begin{array}{c} P_{\text{out}}^{0}=1-P\left(\chi_{2s}^{2}\geq \frac{2\left(s-1\right)\left(1-C_{L}^{0}\right)}{\left(1-H_{1}\right)}|\lambda =\lambda_{0}\right)+P\left(\chi_{2s}^{2}\geq \frac{2\left(s-1\right)\left(1-C_{L}^{0}\right)}{\left(1-H_{2}\right)}|\lambda =\lambda_{0}\right). \end{array}$$

The in-control ARL of the proposed control chart when *C*_*L*_=*C*_*L*_^0^ is denoted by ARL_0_ and given as follows:

(9) $$\begin{array}{c} {\text{ARL}}_{0}=\frac{1}{P_{\text{out}}^{0}}. \end{array}$$

Suppose that the manufacturing process has shifted from *λ*_0_ to *λ*_1_ = *kλ*_0_, where *k* is a shift constant. The probability that the process is declared to be out-of-control when the process is at *λ* = *λ*_1_ is given by

(10) $$\begin{array}{c} P_{\text{out}}^{1}=1-P\left(\chi_{2s}^{2}\geq \frac{2\left(s-1\right)\left(1-C_{L}^{1}\right)}{\left(1-H_{1}\right)}|\lambda =\lambda_{1}\right)+P\left(\chi_{2s}^{2}\geq \frac{2\left(s-1\right)\left(1-C_{L}^{1}\right)}{\left(1-H_{2}\right)}|\lambda =\lambda_{1}\right), \end{array}$$

where *C*_*L*_^1^=1 − *λ*_1_*L*=1 − *kλ*_0_*L*=1 − *k*(1 − *C*_*L*_^0^). (When preparing tables, specify *C*_*L*_^0^ and *k*. Then, *C*_*L*_^1^ can be obtained.)

The ARL for the shifted process is denoted by ARL_1_ and given by

(11) $$\begin{array}{c} {\text{ARL}}_{1}=\frac{1}{P_{\text{out}}^{1}}. \end{array}$$

To construct the proposed control chart for exponential and Weibull distributions based on the lifetime performance index under Type II censoring, we determine the optimal parameters *s* (number of failures to be observed), *H*_1_, and *H*_2_ such that the in-control ARL (ARL_0_) is very close to the specified ARL (say, *r*_0_). In addition, we minimize both ARL_1_ and *s* while finding the optimal parameters since the control chart is considered as effective if it detects the process shift quickly and uses the minimum number of observations to detect the shift. The following optimization problem can be utilized in determining the optimal parameters:

(12) $$\begin{array}{c} \text{minimize}{\text{ARL}}_{1}\;\mathrm{and}\;s\\ \text{subject to}\text{ARL}\geq r_{0},\;n\geq s,\;H_{2}>H_{1}. \end{array}$$

The optimal parameters are determined for two specified in-control ARLs such as 300 and 370, and four different values for the lifetime performance index are considered as *C*_*L*_^0^ = 1.33, 1.50, 1.67, and 2.0 when the process is in-control. For various shift constant values, the out-of-control ARL (i.e., ARL_1_) is calculated using the optimal parameters and the shift constant *k* is taken from 0.9 to 0.1. Tables 1 and 2 provide the out-of-control ARL values along with the optimal parameters, and it should be noted that the performance of the process will decrease when there is a shift in the process. In particular, such performance decreases if there is a decrement in shift. The decreasing trend of out-of-control ARLs is observed from Tables 1 and 2 when the shift value decreases.

### 2.2. Designing of the Proposed Control Chart under Weibull Distribution

Suppose that the random variable *T* follows the Weibull distribution with shape parameter *δ* and scale parameter *θ*. The Weibull distribution is the generalization of the exponential distribution. The pdf of the Weibull distribution is given by

(13) $$\begin{array}{c} f\left(t;\theta ,\delta \right)=\frac{\delta }{\theta }{\left(\frac{t}{\theta }\right)}^{\delta -1}\exp\left(-{\left(\frac{t}{\theta }\right)}^{\delta }\right),\;t\geq 0,\theta >0,\delta >0. \end{array}$$

The mean (*µ*_*T*_) and variance (*σ*_*T*_) of the Weibull distribution are obtained as

(14) $$\begin{array}{c} \mu_{T}=\theta \;\Gamma \left(1+\frac{1}{\delta }\right),\\ \sigma_{T}^{2}=\theta^{2}\;\left[\Gamma \left(1+\frac{2}{\delta }\right)-\Gamma^{2}\left(1+\frac{1}{\delta }\right)\right]. \end{array}$$

The lifetime index for the Weibull distribution is given as

(15) $$\begin{array}{c} C_{L}=\frac{\mu_{T}-L}{\sigma_{T}}=\frac{1}{A}\left[\Gamma \left(1+\frac{1}{\delta }\right)-\frac{L}{\theta }\right]. \end{array}$$

where −*∞* < *C*_*L*_ < Γ(1+(1/*δ*))/*A* and $A=\sqrt{\Gamma \left(1+\left(2/\delta \right)\right)-\Gamma^{2}\left(1+\left(1/\delta \right)\right)}$.

The lifetime-conforming rate *r* is given by

(16) $$\begin{array}{c} r=P\left(T\geq L\right)=\exp\left(-{\left(\frac{L}{\theta }\right)}^{\delta }\right)=\exp\left[-{\left(\Gamma \left(1+\frac{1}{\delta }\right)-AC_{L}\right)}^{\delta }\right]=1-p, \end{array}$$

where *p* is the lifetime-nonconforming rate. In Type II censoring, *s* failures *t*_(1)_, *t*_(2)_,…, *t*_(*s*)_ are noted from *t*_(1)_, *t*_(2)_,…, *t*_(*n*)_. Wu et al. [20] provided the estimator for *C*_*L*_ when *δ* is known under Type II right censoring which is given by

(17) $$\begin{array}{c} {\hat{C}}_{L}=\frac{1}{A}\left[\Gamma \left(1+\frac{1}{\delta }\right)-\frac{L\Gamma \left(s\right)}{D^{1/\delta }\Gamma \left(s-\left(1/\delta \right)\right)}\right], \end{array}$$

where *D*=∑_*i*=1_^*s*^(*n* − *i*+1)(*t*_(*i*)_^*δ*^ − *t*_(*i* − 1)_^*δ*^), and according to Wu et al. [20], for Type II censored data, we have 2∑_*i*=1_^*s*^*Z*_*i*_=2*θ*^−*δ*^*D* ~ *χ*_2*s*_^2^. The probability that the process is declared to be out-of-control is given as in equation (6). Therefore,

(18) $$\begin{array}{c} P_{\text{out}}=1-P\left(\frac{1}{A}\left[\Gamma \left(1+\frac{1}{\delta }\right)-\frac{L\Gamma \left(s\right)}{D^{1/\delta }\Gamma \left(s-\left(1/\delta \right)\right)}\right]\geq H_{1}\right)\\ +P\left(\frac{1}{A}\left[\Gamma \left(1+\frac{1}{\delta }\right)-\frac{L\Gamma \left(s\right)}{D^{1/\delta }\Gamma \left(s-\left(1/\delta \right)\right)}\right]\geq H_{2}\right),\\ P_{\text{out}}=1-P\left(\chi_{2s}^{2}\geq \frac{2{\left[\Gamma \left(1+\left(1/\delta \right)\right)-AC_{L}\right]}^{\delta }\Gamma^{\delta }\left(s\right)}{{\left[\Gamma \left(1+\left(1/\delta \right)\right)-AH_{1}\right]}^{\delta }\Gamma^{\delta }\left(s-\left(1/\delta \right)\right)}\right)\\ +P\left(\chi_{2s}^{2}\geq \frac{2{\left[\Gamma \left(1+\left(1/\delta \right)\right)-AC_{L}\right]}^{\delta }\Gamma^{\delta }\left(s\right)}{{\left[\Gamma \left(1+\left(1/\delta \right)\right)-AH_{2}\right]}^{\delta }\Gamma^{\delta }\left(s-\left(1/\delta \right)\right)}\right). \end{array}$$

The probability that the process is declared to be out-of-control when the process is at *C*_*L*_=*C*_*L*_^0^=(1/*A*)[Γ(1+(1/*δ*)) − (*L*/*θ*_0_)] is given by

(19) $$\begin{array}{c} P_{\text{out}}^{0}=1-P\left(\chi_{2s}^{2}\geq \frac{2{\left[\Gamma \left(1+\left(1/\delta \right)\right)-AC_{L}^{0}\right]}^{\delta }\Gamma^{\delta }\left(s\right)}{{\left[\Gamma \left(1+\left(1/\delta \right)\right)-AH_{1}\right]}^{\delta }\Gamma^{\delta }\left(s-\left(1/\delta \right)\right)}\right)\\ +P\left(\chi_{2s}^{2}\geq \frac{2{\left[\Gamma \left(1+\left(1/\delta \right)\right)-AC_{L}^{0}\right]}^{\delta }\Gamma^{\delta }\left(s\right)}{{\left[\Gamma \left(1+\left(1/\delta \right)\right)-AH_{2}\right]}^{\delta }\Gamma^{\delta }\left(s-\left(1/\delta \right)\right)}\right). \end{array}$$

The in-control ARL of the proposed control chart under Weibull distribution is obtained by using equation (10). Suppose that the manufacturing process has shifted from *θ*_0_ to *θ*_1_ = *kθ*_0_, where *k* is a shift constant. Then, the probability that the process is declared to be out-of-control when the process is at *θ* = *θ*_1_ is given by

(20) $$\begin{array}{c} P_{\text{out}}^{1}=1-P\left(\chi_{2s}^{2}\geq \frac{2{\left[\Gamma \left(1+\left(1/\delta \right)\right)-AC_{L}^{1}\right]}^{\delta }\Gamma^{\delta }\left(s\right)}{{\left[\Gamma \left(1+\left(1/\delta \right)\right)-AH_{1}\right]}^{\delta }\Gamma^{\delta }\left(s-\left(1/\delta \right)\right)}\right)\\ +P\left(\chi_{2s}^{2}\geq \frac{2{\left[\Gamma \left(1+\left(1/\delta \right)\right)-AC_{L}^{1}\right]}^{\delta }\Gamma^{\delta }\left(s\right)}{{\left[\Gamma \left(1+\left(1/\delta \right)\right)-AH_{2}\right]}^{\delta }\Gamma^{\delta }\left(s-\left(1/\delta \right)\right)}\right). \end{array}$$

where *C*_*L*_=*C*_*L*_^0^=(1/*A*)[Γ(1+(1/*δ*)) − (*L*/*θ*_0_)] and *C*_*L*_^1^=(1/*A*)[Γ(1+(1/*δ*)) − (*L*/*θ*_1_)]=(1/*A*)[Γ(1+(1/*δ*)) − (*L*/*kθ*_0_)]. The value of *C*_*L*_^1^ can be obtained from*C*_*L*_^0^ as follows: *C*_*L*_^1^=(1/*A*)(Γ(1+(1/*δ*))(1 − (1/*k*)))+(*C*_*L*_^0^/*k*).

One can obtain the ARL for the shifted process under Weibull distribution using equation (12). Also, the optimization problem given in equation (13) is used to determine the optimal parameters for the proposed control chart construction under Weibull distribution. The optimal parameters are determined under Weibull distribution for the same two specified in-control ARLs such as 300 and 370, and three different values *C*_*L*_^0^ = 1.33, 1.50, and 1.67 are considered as the case of exponential distribution. Here, the out-of-control ARL is calculated for shift constant *k* = 0.95(0.05)0.5. The optimal parameters and the corresponding out-of-control ARL values are reported in Tables 3 and 4. From these tables, it can be understood that the out-of-control ARLs decrease when the shift value decreases. In addition, it is observed that the ARL decreases if there is an increment in the required number of failure items.

## 3. Industrial Application

The contribution of control charts in producing high-reliability products through monitoring and detecting the process variation is an important one. Most of the industrialists have considered that this control chart is one of the useful tools to make the business as profitable. Suppose that the manufacturer of the electronic component wants that the lifetime of producing products should be very high and he decides to use the control chart for process monitoring. The proposed control chart under exponential distribution will be appropriate for monitoring the lifetime since it is considered that exponential distribution is the suitable model to represent the lifetime of electronic components. The performance of the proposed control chart in detecting the process shift is investigated by using simulated data, and data are given in Table 5. Such data have been simulated for exponential distribution, for the following specifications: in-control ARL is 300 (i.e., *r*_0_ = 300) and sample size *n* = 30, and we assume that *C*_*L*_=*C*_*L*_^0^ = 1.67 (i.e., the process is in-control) where the lower limit is *L* = 0.387. The optimal values obtained for these specifications are as follows: *s* = 3, *H*_1_ = 0.108, and *H*_2_ = 1.137. To compute the performance index, the first three failure times of sample items in each of the 10 subgroups is considered, and such index is calculated and plotted in Figure 1. It can be observed from the figure that the performance index of each subgroup lies between decision criteria. Therefore, the process is declared to be in-control. Similarly, we can show the lifetime performance of the process by using simulated data where the lifetime follows Weibull distribution.

## 4. Conclusion

A number of variable-control chart designing methods are available for monitoring the mean, standard deviation, etc. Similarly, some studies are available on designing the control charts for monitoring the performance of the manufacturing process using the capability index. We have also investigated the lifetime performance of the process using one of the capability indices, namely, lifetime performance index with the help of control chart. The designing of the proposed control chart for both the exponential and Weibull distributions has been discussed, and to reduce the time consumption, Type II censoring scheme is used. We have minimized the out-of-control average run length and the number of failure items which are some of the important parameters helpsto decide whether the process is in-control or out-of-control. The performance of the proposed control chart has been explained by using simulated data. It is concluded that the proposed control chart will be very helpful to the manufacturer for monitoring the performance of the process. The proposed chart has the limitation that it can be applied when the lifetime follows the Weibull distribution and cannot be applied for normally distributed data. In this study, designing of the control chart is given for monitoring the lifetime performance of the process where the lifetime follows exponential and Weibull distributions. As a result, there can be a future study on designing control charts for other lifetime distributions and also, an economic designing of the proposed control chart will also be considered.

## Figures and Tables

**Figure 1:** Performance of the proposed control chart.

**Table 1:** ARLs of the proposed control chart under exponential distributions when *r*_0_ = 300.

*k*	*s* = 5, *H*_1_ = 1.000, *H*_2_ = 1.100	*s* = 3, *H*_1_ = 1.000, *H*_2_ = 1.102	*s* = 3, *H*_1_ = 0.108, *H*_2_ = 1.137	*s* = 3, *H*_1_ = 0.932, *H*_2_ = 1.204
	*C*_*L*_^0^ = 1.33	*C*_*L*_^0^ = 1.5	*C*_*L*_^0^ = 1.67	*C*_*L*_^0^ = 2.0
1.0	308.85	307.58	301.88	307.58
0.9	121.01	139.32	137.05	139.32
0.8	49.33	64.35	63.44	64.35
0.7	21.10	30.43	30.07	30.43
0.6	9.59	14.83	14.69	14.83
0.5	4.70	7.51	7.45	7.51
0.4	2.55	4.00	3.98	4.00
0.3	1.57	2.29	2.28	2.29
0.2	1.15	1.45	1.45	1.45
0.1	1.01	1.08	1.08	1.08

**Table 2:** ARLs of the proposed control chart under exponential distribution when *r*_0_ = 370.

*k*	*s* = 5, *H*_1_ = 1.000, *H*_2_ = 1.098	*s* = 4, *H*_1_ = 0.579, *H*_2_ = 1.127	*s* = 5, *H*_1_ = 1.000, *H*_2_ = 1.199	*s* = 3, *H*_1_ = 1.000, *H*_2_ = 1.199
	*C*_*L*_^0^ = 1.33	*C*_*L*_^0^ = 1.5	*C*_*L*_^0^ = 1.67	*C*_*L*_^0^ = 2.0
1.0	375.51	377.22	374.95	376.28
0.9	143.34	154.12	143.16	166.39
0.8	56.94	64.86	56.88	75.03
0.7	23.74	28.31	23.72	34.65
0.6	10.52	12.93	10.51	16.49
0.5	5.04	6.26	5.03	8.16
0.4	2.66	3.27	2.66	4.25
0.3	1.62	1.90	1.61	2.38
0.2	1.16	1.27	1.16	1.48
0.1	1.01	1.03	1.01	1.09

**Table 3:** ARLs of the proposed control chart under Weibull distribution with shape parameter *δ* = 2 when *r*_0_ = 300.

*k*	*s* = 5, *H*_1_ = 0.676, *H*_2_ = 1.612	*s* = 4, *H*_1_ = 0.927, *H*_2_ = 1.714	*s* = 3, *H*_1_ = 1.214, *H*_2_ = 1.808
	*C*_*L*_^0^ = 1.33	*C*_*L*_^0^ = 1.5	*C*_*L*_^0^ = 1.67
1.00	302.64	303.42	306.86
0.95	219.49	237.78	258.95
0.90	143.77	167.78	198.44
0.85	91.24	114.05	146.14
0.80	56.99	76.05	105.40
0.75	35.16	49.91	74.72
0.70	21.47	32.26	52.06
0.65	13.03	20.56	35.60
0.60	7.91	12.94	23.89
0.55	4.84	8.08	15.72
0.50	3.04	5.05	10.15

**Table 4:** ARLs of the proposed control chart under Weibull distribution with shape parameter *δ* = 2 when *r*_0_ = 370.

*k*	*s* = 5, *H*_1_ = 0.644, *H*_2_ = 1.614	*s* = 6, *H*_1_ = 1.088, *H*_2_ = 1.690	*s* = 7, *H*_1_ = 1.457, *H*_2_ = 1.777
	*C*_*L*_^0^ = 1.33	*C*_*L*_^0^ = 1.5	*C*_*L*_^0^ = 1.67
1.00	373.51	370.50	376.73
0.95	271.45	250.85	236.85
0.90	177.09	153.11	135.96
0.85	111.76	90.91	76.45
0.80	69.36	53.30	42.65
0.75	42.46	30.97	23.73
0.70	25.70	17.92	13.26
0.65	15.42	10.39	7.51
0.60	9.23	6.09	4.38
0.55	5.56	3.67	2.68
0.50	3.42	2.32	1.77

**Table 5:** Simulated data for exponential distribution.

1	2	3	4	5	6	7	8	9	10
0.056	0.020	0.016	0.010	0.122	0.021	0.020	0.076	0.015	0.010
0.105	0.037	0.030	0.050	0.137	0.050	0.020	0.081	0.044	0.051
0.143	0.042	0.072	0.056	0.165	0.082	0.125	0.102	0.055	0.060
0.229	0.054	0.257	0.087	0.174	0.098	0.142	0.105	0.064	0.104
0.349	0.078	0.260	0.147	0.285	0.194	0.156	0.112	0.074	0.108
0.387	0.081	0.276	0.172	0.286	0.206	0.221	0.148	0.139	0.111
0.400	0.135	0.278	0.257	0.289	0.254	0.298	0.181	0.160	0.132
0.408	0.166	0.298	0.313	0.294	0.280	0.314	0.281	0.161	0.166
0.428	0.237	0.349	0.339	0.406	0.366	0.330	0.329	0.237	0.206
0.445	0.275	0.467	0.372	0.438	0.397	0.372	0.470	0.255	0.215
0.473	0.286	0.573	0.533	0.463	0.455	0.427	0.509	0.290	0.221
0.531	0.316	0.611	0.580	0.512	0.474	0.510	0.513	0.313	0.286
0.581	0.319	0.625	0.617	0.559	0.561	0.636	0.618	0.338	0.297
0.684	0.327	0.672	0.622	0.783	0.633	0.664	0.622	0.438	0.312
0.724	0.374	0.679	0.818	0.843	0.651	0.666	0.808	0.519	0.338
0.777	0.424	0.875	0.842	0.843	0.652	0.727	0.916	0.545	0.354
0.790	0.527	0.883	0.988	0.933	0.703	0.808	1.036	0.594	0.466
0.797	0.681	1.026	1.021	0.960	0.715	0.906	1.071	0.673	0.498
0.988	0.788	1.056	1.157	1.034	0.758	0.983	1.077	0.751	0.684
1.017	0.816	1.091	1.536	1.044	0.979	1.021	1.089	0.904	0.715
1.061	1.225	1.109	1.567	1.075	1.015	1.044	1.394	0.909	0.937
1.115	1.368	1.148	1.578	1.314	1.213	1.206	1.476	0.993	1.306
1.186	1.434	1.149	1.634	1.331	1.534	1.229	1.481	1.017	1.382
1.386	1.823	1.221	2.757	1.351	1.635	1.290	1.557	1.112	1.488
1.437	1.925	1.248	3.343	1.457	1.640	1.316	1.628	1.244	1.878
1.679	1.980	1.905	3.417	1.760	2.148	1.447	1.690	1.690	2.353
1.852	2.172	1.948	3.541	1.877	2.261	1.775	1.904	2.328	2.413
2.360	3.211	3.054	5.071	2.299	2.571	2.001	2.175	2.345	3.235
2.881	3.233	3.409	5.134	2.380	4.046	2.065	2.279	2.745	3.937
2.948	5.987	4.790	5.317	4.535	4.149	2.379	2.282	5.069	4.114

${\hat{C}}_{L}$									
0.814	0.372	0.625	0.525	0.841	0.673	0.781	0.743	0.516	0.555

## Data Availability

The data are included within the paper.
